# Role of microRNA-15a-5p in the atherosclerotic inflammatory response and arterial injury improvement of diabetic by targeting FASN

This article has been retracted.

**DOI:** 10.1042/BSR20181852

**Published:** 2019-07-02

**Authors:** Yang Liu, Ling-yun Liu, Ye Jia, Yan-yan Sun, Fu-zhe Ma

**Affiliations:** 1 Department of Nephrology, The First Hospital of Jilin University, Changchun 130000, Jilin, P.R. China; 2 Department of Andrology, The First Hospital of Jilin University, Changchun 130000, Jilin, P.R. China; 3 Department of Nephrology, Jilin Province FAW General Hospital, Changchun 130000, Jilin, P.R. China

**Keywords:** Atherosclerotic inflammation, Atherosclerosis, Arterial injury, Diabetes, miR-15a-5p

## Abstract

The present study aims to investigate the mechanism of miR-15a-5p in the atherosclerotic (AS) inflammatory response and arterial injury improvement in diabetic rats by regulating fatty acid synthase (FASN). Initially, bioinformatics tools were applied to evaluate miRNAs and genes correlating with AS, and the target relation between miRNAs and FASN was measured using the Dual-Luciferase Reporter Assay. Subsequently the diabetic AS rat model was established and the surviving rats were divided into: negative control (NC), miR-15a-5p mimic, miR-15a-5p inhibitor, sh-FASN and miR-15a-5p + sh-FASN groups. Then a series of experiments were performed to examine the degree of AS in each group. The results revealed that compared with the NC group, the expressions of C-reactive protein (CRP), interleukin 6 (IL-6), intercellular cell adhesion molecule-1 (ICAM1) in rat arterial tissue, as well as the levels of low-density lipoprotein cholesterol (LDL-C), blood glucose (BG), triglycerides (TG), total cholesterol (TC) and Homocysteine (Hcy) in rat serum, were increased after inhibiting miR-15a-5p, while the level of high-density lipoprotein cholesterol (HDL-C) was decreased and the fat storage area was enlarged after this treatment (*P*<0.05). In the miR-15a-5p mimic and sh-FASN groups, serum HDL-C levels were increased and the fat storage areas in arteries were reduced. The levels of CRP, IL-6, ICAM1 in rat arterial tissue, along with the levels of LDL-C, BG, TG, TC and Hcy in rat serum, were decreased (*P*<0.05). Hematoxylin and Eosin (HE) staining and transmission electron microscopy (TEM) results showed AS lesions to be apparent in the arteries of rats in both the NC and miR-15a-5p inhibitor groups, but that in miR-15a-5p and sh-FASN group were improved, the miR-15a-5p mimic + sh-FASN group showed the most obvious improvement. Taken together, miR-15a-5p alleviates the inflammation response and arterial injury in diabetic AS rats by targeting FASN.

## Introduction

Diabetes is a common disease that can lead to a higher risk of cardiovascular disease (CVD) and certain severe polyvascular complications, including arteriosclerosis and peripheral arterial disease [1,2]. Atherosclerosis (AS), a specific form of arteriosclerosis, is a chronic disease of the arterial wall that represents a main cause for the loss of productivity and increased rates of deaths worldwide [3,4]. AS risk results from several factors, including being of the male gender, having hypertension and family history of illness [5]. The long-term expansion of smooth muscle cells (SMCs) and arterial endothelial cells have been shown to be involved in AS [6]. The structural and functional integrity of the endothelium is crucial in maintaining cardiovascular homeostasis and preventing AS [7]. Dysfunctions of the endothelium and arterial vasculature are primary culprits for atherosclerotic CVD and the progression of AS [8,9].

MicroRNAs (miRs) are a diverse class of highly conserved, small, noncoding RNAs shown to play a critical role in fundamental biological processes, ranging from cell apoptosis and proliferation to cellular differentiation [10]. miRNAs hybridize with complementary sequences in mRNA and silence genes by destabilizing the mRNA or preventing its translation. Over 60% of human protein-coding genes are regulated by miRs [11]. By targeting genetic or other signaling pathways, one member of this family, miR-15a-5p, has been suggested to possibly suppress cell survival and promote apoptosis in certain diseases, such as chronic myeloid leukemia and endometrial cancer cell [12,13]. Fatty acid synthase (FASN), which is directly correlated with the fatty acids synthesis, is a multifunctional protein that plays a central role in *de novo* lipogenesis in mammals [14]. Normally, FASN is expressed highly in several types of human tumors, while existing at lower levels in normal tissues. Thus, the inhibition of the FASN gene has been proven to be effective in suppressing cell proliferation [15]. High expression of the FASN gene could lead to proliferation and migration of endothelial cells [16]. Given that the migration of vascular endothelial cells plays an important role in AS, miR-15a-5p is predicted to target FASN. Hence, the present study aims to investigate the mechanism of miR-15a-5p targeting FASN in AS arterial tissue.

## Materials and methods

### Model establishment

Forty specific pathogen-free (SPF) male apolipoprotein E gene-knockout (Apoe^−/−^) rats (aged 8 weeks, Art. No. J003, Nanjing Better Biotechnology Co., Ltd, Nanjing, China) were randomly divided into the model group (*n*=35) and the control group (*n*=5). Fasting blood glucose (FBG) levels were detected after the rats had been adaptively fed for 1 week. After 12 h of fasting, the rats in model group were continuously injected intraperitoneally with 55 mg/kg buffer solution containing streptozotocin (STZ) for 5 days, while rats in the control group were injected with STZ-free buffer solution, the other procedures were carried out with no difference with that of model group. The FBG levels in the rats at the last time of injection and at 10 days after injection were detected from blood extracted from the rats’ eyeballs. The models were deemed successfully established if the level of FBG was up to 11.1 mmol/l [17].

### Carrier construction

The mRNA sequence for FASN was obtained from the National Center for Biotechnology Information (Accession number: NM _007988). The corresponding shRNA and negative control (NC) sequences were designed using BLOCK-iT™ RNAi Designer (http://rnaidesigner.thermofisher.com/rnaiexpress) and synthesized by Shanghai Genechem Co., Ltd. (Shanghai, China.) The sequences were then cloned to the plasmid vector pcDNA3.1 (VPI0001, Invitrogen) containing restriction sites HindIII and XHoI. After an hour of connection at 16°C, the products were added into competent *Escherichia coli* DH5α (D9052, Takara) for transformation. The resistant bacterial colony was then identified and selected by means of enzyme digestion and polymerase chain reaction (PCR). Subsequently, the plasmids were quickly extracted and preserved at −20°C, and then transfected into the rat hepatocytes (IAR20, Shanghai Jining Shiye Industrial Co,. Ltd. Shanghai, China). Expression of FASN mRNA in rat hepatocytes was measured using quantitative reverse-transcription PCR (qRT-PCR); the sequence with best interference was chosen for the following experiment.

### Dual-luciferase reporter assay

Potential miRNAs which could regulate FASN expression were measured using miRNA–mRNA relationship prediction websites, including TargetScan (http://www.targetscan.org/vert_71/), miRDB (http://34.236.212.39/microrna/getGeneForm.do), miRWalk (http://mirwalk. umm.uni-heidelberg.de/) and miRsearch (https://www.exiqon.com/miRSearch). The results obtained from these websites were compared using the online Venn diagram analysis tool, Venny2.1 (http://bioinfogp.cnb.csic.es/tools/venny/index.html). Next, the FASN 3′UTR wild-type sequence (FASN 3′UTR-wt) and the site-directed mutagenesis sequence toward miRNA binding site FASN 3′UTR-mut were designed. This was followed by construction of the luciferase reporter carrier and transfecting Chinese hamster ovary (CHO) cells (Art. No. CC-Y2110, ATCC, U.S.A.). Luciferase activity in the samples was detected by Dual-Luciferase Reporter Assay. Forty-eight hours after transfection, the used medium was discarded and the samples were washed with phosphate-buffered saline (PBS) twice. To the cells of each well, 100 μl of Passive Lysis Buffer (PLB) were added and mixed for 15 min, after which the cell lysate was collected. Subsequently, the LARStop&Glo® Reagent was applied to detect luciferase with the pre-measure time set to 2 s, measure time set to 10 s, and the sample added at each time set to 100 μl. Twenty microliters of each cell lysate was added to the luminotron, and the activity of luciferase was detected using the bioluminescence detector (VersaMax M3, Molecular Devices, U.S.A.). The experiment was repeated three times.

### Animal grouping and transfection

The successfully modeled and surviving rats were further divided into the NC group (rats injected with NC sequence mediated by liposome through caudal vein), the miR-15a-5p mimic group (rats injected with miR-15a-5p mimic), the miR-15a-5p inhibitor group (rats injected with miR-15a-5p inhibitor), sh-FASN group (rats injected with sh-FASN recombinant plasmid), miR-15a-5p mimic + sh-FASN group (rats injected with miR15a-5p mimic and sh-FASN recombinant plasmid). Injections were made following the instructions for Lipofectamine 2000: 0.5 μl of shRNA was added into tube 1 (miR mimic or inhibitor, concentration at 2 μg/μl); 0.55 μl of Lipofecatmine and 0.45 μl of RNase-free water were added into tube 2. After mixing the contents of two tubes for 30 min at room temperature, the resulting mixture was injected into the caudal veins of the rats at a concentration of 0.2 ml/10g.

### Materials collection

Four weeks after grouping, the rats were anesthetized by intraperitoneal injection with 3% Nembutal (30 mg/kg) and then killled. The bodies were disinfected in 75% ethanol for 3 min and then fixed on a table. The rats’ peripheral blood was collected and separated (3000 r/min, 4°C), and the serum was then preserved at −80°C. Following removal of the skin and muscles covering the rats’ chests and abdomens, thoracic and abdominal aortas were collected and preserved at −80°C.

### qRT-PCR

The preserved aortic tissues were ground and centrifuged in liquid nitrogen. The total RNA of the arterial tissues was extracted in accordance with kit instructions. After extraction, the optical density (OD) at 260 and 280 nm of each RNA sample was measured using an ND-1000 spectrophotometer, and the RNA concentration was adjusted for the following experiments. Reverse transcription of the cDNA was conducted using the two-step method in accordance with kit instructions. The reaction conditions were set as follows: 70°C for 10 min, ice bath for 2 min, 42°C for 60 min, and 70°C for 10 min. The cDNA was stored at −80°C for a short time and then served as a template for q-PCR. q-PCR was conducted using the miScript SYBR Green PCR Kit (Qiagen Company, Valencia, CA), and the reaction sequences are shown in Table 1. Following the instructions of reaction system, 25 μl of overall reaction liquid was confected: 2× QuantiTect SYBR Green PCR 12.5 μl, 10× miscript Primer Assay 140/27a/U6 2.5 μl, RNase-free water 7.5 μl and Template cDNA for 2.5 μl, with three wells set for each sample. Forty cycles were conducted with reaction conditions as follows: pre-denaturation at 95°C for 15 min; denaturation at 94 °C for 15 s; cooling at 55°C for 30 s; extension at 70°C for 30 s. Detection was made using a 7300 PCR kit (Applied Biosystems, Inc., CA, U.S.A.). U6 was used as the internal control for miRNA, while β-actin was set as the internal control for other genes. Melting curves were used to evaluate the reliability of the PCR results, and the specificity of primers was judged by the melting curves of the products. The relative mRNA expression of target gene was calculated based on the 2^−ΔΔ*C*^_t_ method [18]. Each experiment was repeated three times; Δ*C*_t_ (threshold cycle) refers to the difference value between target genes and internal control genes.

**Table 1:** Primer sequences for qRT-PCR

Gene	Forward (5′–3′)	Forward (5′–3′)
*Fasn*	AGCACTGCCTTCGGTTCAGTC	AAGCGCTGTGGAGGCCACTTG
*CRP*	TTTCGCTAGCATGGAGAAGCTACTCTGG	GAACGAATTCTCAGGACCACAGCTGCG
*IL-6*	TGGAGTCACAGAAGGAGTGGCTAAG	TCTGACCACAGTGAGGAATGTCCAC
*ICAM1*	AGGTGTGATATCCGGTAGAT	CCTTCTAAGTGGTTGGAACA
*β-actin*	AGGGAAATCGTGCGTGACATTAAA	ACTCATCGTACTCCTCCTTGCTGA
*miR-15a-5p*	GGGTAGCAGCACATAATGGTTTGTG	CAGTGCGTGTCGTGGAGT
*miR-92a-2-5p*	GGGAGGTGGGGATTGGUGGCATTAC	CAGTGCGTGTCGTGGAGT
*U6*	GTGCTCCTGCTTCGGCAGCACATATAC	CGTTGACATCCGTAAAGAC

### Western blot

Tissue samples and RIPA lysis buffer (P0013C, Beyotime Biotechnology Co., Shanghai, China) were placed in centrifuge tubes and centrifuged at 12000 rpm at 4°C for 10 min. The supernatant was then collected and diluted for protein quantitation. Loading buffer was added to adjust the concentrations and volumes of tissue proteins. Twenty micrograms of the samples was placed in each well, and the protein was separated using electrophoresis with 12% polyacrylamide gel. After electrophoresis and transferring to PVDF membranes, the proteins of samples were sealed on a decolorization shaker by Tris-buffered solution + Tween (TBST) containing 5% bovine serum albumin (BSA) for 1 h at room temperature. Following discarding of the blocking and placement of the membrane into the plastic groove, the samples were treated with C-reactive protein (CRP) primary antibodies (Art. No. ab46820, diluted at 1:2000–5000), Interleukin 6 (IL-6, Art. No. ab208113, diluted at 1:1000), intercellular cell adhesion molecule-1 (ICAM1, Art. No. ab119871, diluted at 1:1000) and β-actin (Art. No. ab8227, diluted at 1:1000–5000) and kept overnight at 4°C. On the following day, the samples were washed three times with TBST for 10 min each. The samples were then treated with horseradish peroxidase (HRP)-labeled secondary antibody IgG (Art. No. ab205718, diluted at 1:2000–5000) and incubated at room temperature for 1 h. All antibodies were provided by Abcam Inc., Cambridge, MA, U.K. Next, the samples were further washed with TBST three times for 5 min each, colored using Electrochemiluminescence (ECL), exposed with X-ray radiation and imaged. The E-Gel Imager System (Art. No. 4466613, Thermo Fisher Scientific Inc., Waltham, MA, U.S.A.) was applied for analysis of the absorbance of the colored bands. The relative volume of sample protein was evaluated as: average absorbance of sample/average absorbance of internal control × 100%. The relative volume of each sample protein was compared using statistical analysis. The experiment was repeated three times.

### Enzyme-linked immunosorbent assay

The rats’ BG, high-density lipoprotein cholesterol (HDL-C), low-density lipoprotein cholesterol (LDL-C), triglycerides (TG), total cholesterol (TC) and Homocysteine (Hcy) levels were evaluated using enzyme-linked immunosorbent assay (ELISA) kits purchased from Shanghai Chuangxiang Biotech Company (Shanghai, China). The procedures employed were as follows: a 12-well plate was put in an aluminium foil bag at room temperature for 20 min and then removed, after which the standard wells and sample wells were set. To each standard well, 50 μl of standard product at varying concentrations was added, while the sample well was filled with 10 μl of rat serum and 40 μl of sample diluent. To each well, 100 μl HRP-labeled detection antibody were added and then incubated at 37°C for 50 min. Next, the liquid was discarded and the samples were washed with PBS five times. Fifty microliters of substrates A and B were then added to each well, and the plate was incubated at 37°C for 15 min in the dark. Fifty microliters of stop buffer as added, and, finally the OD value at 450 nm was evaluated.

### Immunohistochemistry

Frozen artery tissues were cut into slices, and the high-pressure method was then for antigen repair. After repairing for 90 s, the slices were cooled to room temperature and washed with PBS for 3 × 3 min. Subsequently 100 μl of 5% BSA were added to the slices, and they were incubated at 37°C for 30 min. The slices were then sealed using anti-CRP (Art. No. ab46820, diluted as 1:2000–5000, Abcam Inc., Cambridge, MA, U.K.) and incubated at 4°C overnight. Next, the slices were washed with PBS, and signed second antibody goat-anti-rabbit was added (HY90046, Shanghai Hengyuan Biotech Company, Shanghai, China) and diluted at 1:100 for 30 min. After washing with PBS, streptavidin-peroxidase (Beijing Zhongshan Biotech Co., Ltd., Beijing, China) was added to the slices, and they were incubated at 37°C for 30 min. The samples were then washed with PSB three times for 3 min each, after which they were stained using diaminobenzidine (DAB, Bioss Biotech, Beijing, China). Next, the slices were soaked in Hematoxylin for 5 min, then washed with tap water, further soaked in 1% hydrochloric acid for 4 s, and washed with water 20 min to return to blue. Finally, the slices were observed under high power lens, and the rate of positively stained area was analyzed.

### Hematoxylin and Eosin staining

The frozen aortic roots were soaked and washed with normal saline, after which the peripheral connective tissue was cleaned. The samples were then fixed in 10% formaldehyde, embedded in paraffin and cut into 5-μm slices. The standard Hematoxylin and Eosin (HE) staining was applied as follows: the embedded slices were successively dewaxed in xylene I (CAS No. 14936-97-1, Shanghai E-Research Biotech Co., Ltd. Shanghai, China) and xylene II (CAS No. 523-67-1, Shanghai Yuduo Biotech Company, Shanghai, China) for 5 min. Following this, the slices were dewaxed for 1 min using 100, 95, 80, 75% ethanol, respectively, and then washed for 2 min using distilled water. Next, the slices were stained using Hematoxylin (CAS No.474-07-7, Qingdao Jisskang Biotechnology Co., Ltd. Qingdao, China) for 5 min and then washed with water. The slices were continuously differentiated in 1% hydrochloric acid and ethanol for 1.5 min and then soaked in warm water for 5 min. After these processes, Eosin staining was applied to these slices (Art. No. RY0648, Qingdao Jisskang Biotechnology Co., Ltd. Qingdao, China) for 2 min, and slices were then washed with water. The above procedures were repeated if no satisfactory result was found. Then the staining results were observed under microscope. After staining, the samples were dehydrated using 95% and 100% methanol for 1 min, then cleaned using dimethylbenzene carbonic acid (3:1), xylene I and xylene II for 1 min. Following air drying, the samples were sealed using resinene. The nuclei showed a deep blue while, the cytoplasm and the fibrous tissues showed red at various degrees.

### Oil Red O staining

The arterial samples were fixed in a formalin calcium solution for 2–3 days and completely washed. After this, the samples were soaked in 60% avantin for 10 min, stained with Oil Red O solution for 3–4 h, and then differentiated using 60% avantin six to seven times. Images were taken using light microscopy (AMEX1000, Thermo Fisher, U.S.A.), and the software, ImageJ, was applied for measuring the total area of fatty streaks within the aorta. The percentage of fatty streak area of the total aortic area was thus evaluated.

### Transmission electron microscopy

The frozen arterial tissues were successively fixed with 2.5% glutaraldehyde, washed with 0.1 mol/l PBS, fixed with 1% osmic acid and washed with 0.1 mol/l PBS again. Following this, the samples were dehydrated using ethanol of different concentrations, embedded, fixed and cut into slices, then observed using a H-9500 TEM (Hitachi Limited, Japan), and images were taken.

### Statistical analysis

The Statistical Package for the Social Sciences (SPSS) 21.0 (SPSS Inc., Chicago, IL, U.S.A.) was applied for data analysis. Categorical data were expressed as mean ± standard deviation (x ± s), and all experiments were repeated for no less than three times. Differences between each group pair were evaluated using the *t* test while the differences among multiple groups were compared using one-way analysis of variance (ANOVA). The normality test was conducted using the Kolmogorov–Smirnov method. Normally distributed data among multiple groups were compared using one-way ANOVA with Tukey’s post-hoc tests, while skewed data distributed among multiple groups were analyzed using Dunn’s multiple comparison for post-hoc tests following Kruskal–Wallis testing. *P*<0.05 was considered to show a statistically significant difference, and *P*<0.01 was considered to show an extremely statistically significant difference.

## Results

### Target regulating relationship between miR-15a-5p and FASN

According to the miRNA–mRNA relationship predicted by web tools including TargetScan, miRDB, miRsearch and MiRWalk, respectively 214, 28, 24 and 3233 miRNAs were shown to have a target relation with the FASN gene. Differences between the miRNAs were compared then using Venn Diagrams. It was shown that mmu-miR-15a-5p and mmu-miR-92a-2-5p are at an intersection point (Figure 1A). miR-15a has been proved to be expressed at lower levels, and to inhibit inflammation and angiogenesis in diabetic retinopathy [19]. On the other hand, miR-92a was shown to be highly expressed in diabetes, while it indirectly promotes the production of Hcy and stimulates the incidence of AS [20,21]. The results of qRT-PCR showed that, compared with control group, miR-15a-5p expression in the model group was lower, while the miR-92a-2-5p and FASN mRNA expressions were higher (Figure 1C), which is in agreement with the results of [20,21]. Normally, miRNA down-regulates gene expression [22]. Hence miR-15a-5p was chosen for this study, and its binding site with FASN was predicted (Figure 1B). The results of the fluorescein reporter suggested that, compared with the cells co-transfected with miR-15a-5p NC and FASN-3′-UTR-wt plasmids, the activation of luciferase in cells co-transfected with miR-15a-5p mimic and Fasn-3′-UTR-wt plasmid was significantly lower (*P*<0.05), while little difference was shown among other groups (all *P*>0.05) (Figure 1D).

**Figure 1:** Target relation between miR-15a-5p and FASN (**A**) mmu-miR-15a-5p and mmu-miR92a-2-5p are shown in intersection according to the miRNA targets for FASN prediction from TargetScan, miRDB, miRsearch and MiRWalk. (**B**) Targeting binding site of miR15a-5p and FASN. (**C**) mRNA expressions of miR-15a-5p, miR-92a-2-5p and FASN in rat arterial tissues. (**D**) miR-15a-5p targets FASN detected by luciferase reporter assay. Data shown are mean ± SD, experiments had been repeated three times, ^#^, *P*<0.05 compared with Control group; &, *P*<0.05 compared with cells cotransfected with miR-15a-5p NC and FASN-3′-UTR-wt plasmid.

### shRNA2 interfered with the greatest efficiency

The expressions of FASN in rat hepatocytes transfected with different FASN-interfering sequences were detected using qRT-PCR. The results demonstrated that, compared with the NC sequence, the mRNA expressions of FASN of other sequences were obviously decreased, and the shRNA2 sequence had the greatest silencing efficiency (all *P*<0.05) (Figure 2). Thus, shRNA2 was chosen for the experiments which followed.

**Figure 2:** Selection of best-interfering shRNA sequence Data shown are mean ± SD, experiments had been repeated three times, *, *P*<0.05 compared with NC group; ^∧^, *P*<0.05 compared with shRNA2 group.

### Overexpression of miR-15a-5p or silencing of FASN suppressed CRP, IL-6 and ICAM1 expressions in rat arterial tissues

The biomarkers for AS in the rats were detected using qRT-PCR and Western blotting, and immunohistochemistry was applied to determine the location and ratio of CRP. The results suggested that CRP is expressed both in the nucleus and endochylema of vascular endothelial cells, SMCs and desmocytes, but mainly in endochylema. Compared with the NC group, CRP, IL-6 and ICAM1 expressions were significantly higher in the miR-15a-5p inhibitor group, and lower in the miR-15a-5p mimic and sh-FASN groups. The above indicators changed more overtly when joint treatment was applied (Figures 3 and 4) (all *P*<0.05).

**Figure 3:** Expressions of CRP, IL-6 and ICAM by qRT-PCR and Western blotting Tail veins of STZ-induced model (n=30 and 5 mice died or were not successfully modeled during STZ induction) rats were injected with liposomes containing different sequences (miR-15a-5p mimic, miR-15a-5p inhibitor or FASN shRNA) threee times a week for 4 weeks. After 4 weeks, the thoracic aortas of each group (n=6 for each group) of rats was isolated and used to detect the expression of CRP, IL-6 and ICAM. (**A**) mRNA expressions of CRP, IL-6 and ICAM; (**B**) band patterns of Western blot of CRP, IL-6 and ICAM. (**C**) Protein expressions of CRP, IL-6 and ICAM. *, *P*<0.05 compared with NC group. Data shown are mean ± SD, experiments had been repeated three times, ^@^, *P*<0.05 compared with miR-15a-5p mimic + sh-FASN group.

**Figure 4:** CRP expression by immunohistochemistry Tail veins of STZ-induced model rats (n=30 and 5 mice died or were not successfully modeled during STZ induction) were injected with liposomes containing different sequences (miR-15a-5p mimic, miR-15a-5p inhibitor or FASN shRNA) three times a week for 4 weeks. After 4 weeks, the thoracic aortas of each group rats (n=6 for each group) was isolated and used for making paraffin slices and immunohistochemical staining. (**A**) Staining image from immunohistochemistry of CRP (400×); (**B**) area percentage of positive CRP. Data shown are mean ± SD, experiments had been repeated three times, *, *P*<0.05 compared with NC group; ^@^, *P*<0.05 compared with miR-15a-5p mimic + sh-FASN group.

### Overexpression of miR-15a-5p or silencing of FASN down-regulated levels of LDL-C, TC, BG, TG, Hcy in rat serums except HDL-C

ELISA results showed that, compared with the NC group, the concentrations of LDL-C, TC, BG, TG and Hcy in rats of the miR-15a-5p inhibitor group increased, while the concentration of HDL-C decreased. Meanwhile, in the miR-15a-5p mimic and sh-FASN groups, the concentrations of LDL-C, TC, BG, TG and Hcy significantly decreased, while the concentration of HDL-C increased (all *P*<0.05) (Table 2 and Figure 5). These results suggested that overexpression of miR-15a-5p or silencing of FASN could ameliorate the indexes of BG and blood lipids.

**Figure 5:** Concentrations of HDL-C, LDL-C and TC in rat serum by ELISA Tail veins of STZ-induced model rats (n=30 and 5 mice died or were not successfully modeled during STZ induction) were injected with liposomes containing different sequences (miR-15a-5p mimic, miR-15a-5p inhibitor or FASN shRNA) three times a week for 4 weeks. After 4 weeks, whole blood is used to isolate serum (n=6 for each group) and HDL-C, LDL-C and TC were quantitated by ELISA**.** Data shown are mean ± SD, experiments had been repeated three times; *, *P*<0.05 compared with NC group; ^@^, *P*<0.05 compared with miR-15a-5p mimic + sh-FASN group.

**Table 2:** Concentrations of BG, TG and Hcy in rat serum according to ELISA

Group	BG (mmol/l)	TG (μmol/l)	Hcy (μmol/l)
NC (*n*=5)	13.1 ± 2.64	2.18 ± 0.10	20.4 ± 2.21
miR-15a-5p mimic (*n*=5)	9.8 ± 0.24*,^†^	1.67 ± 0.20*,^†^	16.3 ± 1.21*,^†^
miR-15a-5p inhibitor (*n*=5)	18.1 ± 2.16*	2.57 ± 0.29*	26.8 ± 2.13*
sh-Fasn (*n*=5)	11.1 ± 1.65*,^†^	1.78 ± 0.65*,^†^	17.6 ± 1.20*,^†^
miR-15a-5p mimic+ sh-Fasn (*n*=5)	8.1 ± 0.40*	1.33 ± 0.5*	13.4 ± 1.02*

*, *P*<0.05 compared with NC group. ^†^, *P*<0.05 compared with miR-15a-5p mimic + sh-Fasn group.

### Overexpression of miR-15a-5p or silencing of FASN improved the pathological conditions of AS rat vasculature

HE staining results (Figure 6) showed the appearance of a large number of inflammatory cells in the arterial tissues of the NC and miR-15a-5p inhibitor groups, while intimal cells proliferated and some cells were broken or had vanished, with a large number of foam cells and fat vacuoles. Moreover, the SMCs of the media proliferated with disorder, demonstrating the pathological conditions of AS. But in the miR-15a-5p mimic and sh-FASN groups, the situation was much improved. The arterial intima was complete and flat, and the SMCs of the media were arranged in an orderly manner without adipocytes or inflammatory cell infiltration.

**Figure 6:** HE staining of rat arterial tissues (200×) Tail veins of STZ-induced model rats (n=30 and 5 mice died or were not successfully modeled during STZ induction) were injected with liposomes containing different sequences (miR-15a-5p mimic, miR-15a-5p inhibitor or FASN shRNA) three times a week for 4 weeks. After 4 weeks, the thoracic aortas of each group rats (n=6 for each group) were isolated and used for making paraffin slices and HE staining.

### Overexpression of miR-15a-5p or silencing of FASN reduced the fat storage of rat arteries

The results of Oil Red O staining demonstrated that, compared with the NC group, the fat storage area was larger in the miR-15a-5p inhibitor group while smaller in the miR-15a-5p mimic and sh-FASN groups (Figure 7). This suggests that overexpression of miR-15a-5p or silencing of FASN could effectively decrease the fat storage area of rat arteries (all *P*<0.05).

**Figure 7:** Oil Red O staining of rat arterial tissues Tail veins of STZ-induced model rats (n=30 and 5 mice died or were not successfully modeled during STZ induction) were injected with liposomes containing different sequences (miR-15a-5p mimic, miR-15a-5p inhibitor or FASN shRNA) three times a week for 4 weeks. After 4 weeks, the thoracic aortas of each group rats (n=6 for each group) was isolated and used for Oil Red O staining. (**A**) Staining image of Oil Red O staining; (**B**) area percentage of fatty streaks. Data shown are mean ± SD, experiments had been repeated three times, *, *P*<0.05 compared with NC group; ^@^, *P*<0.05 compared with miR-15a-5p mimic + sh-FASN group.

### Overexpressed miR-15a-5p or silenced FASN improved the pathological ultrastructure of rat vasculature

Transmission electron microscopy (TEM) results showed that, the endothelial cells of in NC group and the miR-15a-5p inhibitor group were difficult to distinguish, and a large number of vacuoles were generated in the tissues, and a large number of lipid droplets (triangle) were generated in the vacuoles. There were many round holes with different sizes on the surface of intima, which were similar to worm-eaten damage. In miR-15a-5p mimic group and miR-15a-5p inhibitor + sh-FASN group, some vacuoles containing lipid droplets also existed, but the arrangement of endothelial cells could be distinguished to a certain extent. The intima of the aorta in the sh-FASN group was smooth, and the endothelial cells were elongated and arranged parallel to each other. No obvious vacuoles were observed (Figure 8).

**Figure 8:** Ultrastructure of rat arterial tissues (10^4^×) Tail veins of STZ-induced model rats (n=30 and 5 mice died or were not successfully modeled during STZ induction) were injected with liposomes containing different sequences (miR-15a-5p mimic, miR-15a-5p inhibitor or FASN shRNA) three times a week for 4 weeks. After 4 weeks, the thoracic aortas of each group rats (n=6 for each group) was isolated and fixed by osmium acid. The triangles represent lipid droplets; diamonds represent autophagosomes.

## Discussion

Atherosclerotic CVD has become the leading diabetes complication, accounting for almost 70% of mortality in diabetes patients [23]. Moreover, CVD and diabetes share many common pathophysiological characteristics such as insulin resistance, inflammation, high blood pressure and obesity [24–27]. Numerous studies have shown that miRNA can participate in the pathological process of Type 2 DM and CVD by regulating the functions of myocardial cells, vascular SMCs, endothelial cells and platelet cells, inflammatory responses and lipid metabolism pathways. The results of the present study have demonstrated that the expression of miR-15a-5p could target the FASN gene [28]. The results of this study demonstrated that miR-15a-5p can improve AS in mice from two aspects that it can reduces the inflammatory response of endothelial cells and accelerates lipid metabolism by targeting FASN.

The experiments of the present study showed that miR15a-5p closely regulates the expression of FASN. Importantly, it was suggested that the expressions of CRP, IL-6 and ICAM1 were elevated in diabetic AS rats. Moreover, overexpression of miR-15a-5p could reduce the levels of CRP, IL-6 and ICAM1. CRP is a sensitive biomarker for systemic inflammation, and high levels of CRP appeared in every inflammatory state. Increased CRP levels normally indicate a higher risk for several degenerative disorders, such as CVD and diabetes [29]. Previous studies have shown that cells of the arterial wall can locally produce and express CRP, which might in turn be a relevant pro-atherothrombotic stimulus [30,31]. At the same time, CRP is a generally accepted CVD risk marker, and could promote ICAM expression in endothelial cells and stimulate monocyte-endothelial cell adhesion [32]. Another study has demonstrated that the treatment of endothelial cells statins is able to modulate the expression of cell adhesion molecules, such as ICAM1, which emphasize the correlation between ICAM1 and angiocardiopathy [33]. IL-6 levels have been shown to be independently correlated with subclinical atherosclerotic lesions, and this correlation might result from the influence of IL-6 on ICAM1 secretion [34]. Moreover, in the miR-15a-5p mimic and sh-FASN groups, HDL-C levels in rat sera were improved, and arterial fat storage areas were reduced. Meanwhile, the levels of LDL-C, BG, TG, TC and Hcy in rat sera were decreased. An obvious increase in the concentrations of LDL-C and TG has been found in AS patients, while the levels of HDL-C were found at a lower level in these patients. LDL-C has been considered an important risk factor for AS and coronary disease, and the LDL-C/HDL-C has been identified as an marker of AS [35,36]. Thus, the results of this study suggest that the expression of miR-15a-5p and silencing FASN could decrease the inflammatory response in diabetic AS rats.

Importantly, in NC and miR-15a-5p inhibitor group rats, the pathological morphology of AS was clearly seen in arterial tissues and vascular endothelia. A large number of inflammatory cells appeared, while intimal cells proliferated and some cells were broken or had vanished, with the appearance of a large number of foam cells and fat vacuoles. Moreover, SMCs of the media proliferated with disorder. Besides this, endothelial cells of the rats’ vasculature had vanished, became edematous or appeared with necrotic with loose cytoplasms. Vascular cell apoptosis, a form of cell death, plays a crucial role in developing AS, and thus in promoting CVD [37]. High levels of cell apoptosis may lead to endothelial dysfunction, which is a key event in the progression of AS [38,39]. These results demonstrated that a high expression of miR-15a-5p contributes to improvement in function of endothelial cells and lipid metabolism in the arterial tissues of diabetic AS rats.

In summary, the present study provided evidence that overexpression of miR-15a-5p could reduce the inflammation of arterial tissues and vascular endothelial cells and promote lipid metabolism in diabetic AS rats. Overexpressed miR-15a-5p combined with silence of FASN results in a lower level of AS biomarkers, including LDL-C, BG, TG and TC, and decreases the expressions of CRP, IL-6 and ICAM1 in rat serum. All of the experimental results strongly suggest that the increased expression of miR-15a-5p might offer a protective role in the therapies and treatments for patients with AS (Figure 9). In the future, the regulatory mechanism of miR-15a-5p on the course of diabetes mellitus complicated with AS will be explored from other perspectives, such as function of vascular SMC and platelet activity.

**Figure 9:** The potential molecular mechanisms that miR-15a-5p could improve diabetic AS by down-regulating FASN levels miR-145 inhibits the levels of AS biomarkers through targeting FASN. Diabetic AS is improved with overexpression of miR-15a-5p.

## Abbreviations

ANOVA: analysis of variance
AS: atherosclerosis
BG: blood glucose
BSA: bovine serum albumin
CRP: C-reactive protein
CVD: cardiovascular disease
ELISA: enzyme-linked immunosorbent assay
FASN: fatty acid synthase
FBG: fasting blood glucose
Hcy: homocysteine
HDL-C: high-density lipoprotein cholesterol
HRP: horseradish peroxidase
ICAM1: intercellular cell adhesion molecule-1
IL-6: interleukin 6
LDL-C: low-density lipoprotein cholesterol
miR: microRNA
NC: negative control
OD: optical density
PBS: phosphate-buffered saline
PCR: polymerase chain reaction
PLB: Passive Lysis Buffer
qRT-PCR: quantitative reverse-transcription PCR
SMC: smooth muscle cell
STZ: streptozotocin
TBST: Tris-buffered solution + Tween
TC: total cholesterol
TG: triglyceride
